The article "Relationship between proteinuria and optical coherence tomographic features of the chorioretina in patients with pre-eclampsia" was published in 2021. Journal: PLoS One.

# Relationship between proteinuria and optical coherence tomographic features of the chorioretina in patients with pre-eclampsia

**DOI:** 10.1371/journal.pone.0251933

**Published:** 2021-05-20

**Authors:** Kyu Young Shim, Jin Gon Bae, Jae Kyoung Lee, Yu Cheol Kim

**Affiliations:** 1 Department of Ophthalmology, Keimyung University School of Medicine, Daegu, Korea; 2 Department of Obstetrics, Keimyung University School of Medicine, Daegu, Korea; University of Florida, UNITED STATES

## Abstract

This retrospective study aimed to evaluate the correlation between ophthalmologic factors and proteinuria in patients with pre-eclampsia using swept-source optical coherence tomography (OCT) and OCT angiography. In total, 61 pregnant patients diagnosed with pre-eclampsia were recruited during their hospital stay. The authors investigated the relationship between urine protein–creatinine ratio (PCR) and chorioretinal measurements including choroidal thickness (CT), choroidal vascularity index (CVI), foveal avascular zone (FAZ), vascular density (VD), ganglion cell layer+ (GCL+) and GCL++. The associations between mean arterial pressure (MAP) and ophthalmologic factors were also evaluated. Central subfield CT of the right eye (*p* = 0.031) and paracentral CT of both eyes were related to higher PCR (≥1.35 mg/mg). A significant association with PCR after logarithm transformation was noted (*r* = 0.284, *p* = 0.026). Retinal measurements (FAZ, VD, GCL+ and GCL++) and CVI were not related with PCR. There was a positive association between MAP and PCR after logarithm transformation (*r* = 0.296, *p* = 0.021); however, chorioretinal factors were not related with MAP. In pregnant women with pre-eclampsia, CT using OCT is a novel factor that is correlated with PCR. Ocular structural alteration in patients with pre-eclampsia may be one of systemic vascular changes caused by pre-eclampsia rather than hypertension.

## Introduction

Pregnant women undergo adaptive changes in the endocrine, immune and cardiovascular systems to provide an adequate supply for foetus [1–3]. Pre-eclampsia is a pregnancy-specific multisystemic disorder with changes in systemic vascular endothelial cell and haemodynamics arising from placental ischaemia, leading to hepatic failure, proteinuria, neurologic symptom and pulmonary oedema [4,5]. Approximately 30%–40% of patients with pre-eclampsia have subjective visual disturbance; various ocular findings are observed [6,7]. High vascular density (VD) and fenestrated capillaries of the choroid make it sensitive to systemic changes. An imbalance of circulating anti-angiogenic factors including soluble fms-like tyrosine kinase 1 (sFLT1) and angiogenic factors such as vascular endothelial growth factor (VEGF) plays a role in endothelial dysfunction in patients with pre-eclampsia, which in turn influences ocular environment, especially choroid [8–10].

The limitation in penetrance of the previous optical coherence tomography (OCT) hindered in acquiring refined and accurate resolution of the choroid. Recently, the advancement in enhanced depth imaging (EDI) technique or swept-source OCT (SS-OCT) can visualise choroid with higher resolution [11–13]. The advent of OCT angiography (OCT-A) provides vascular distribution of the retina and choroid in a non-invasive method [14,15].

Proteinuria is one of the pivotal features of pre-eclampsia. The spot (random) urine protein–creatinine ratio (normal range PCR, <0.3 mg/mg) was considered an alternative, quick and reliable method to assess quantitative proteinuria [16]. The relationship between serologic and haemodynamic changes of patients with pre-eclampsia and ocular characteristics has been focused by many researchers, but it has not been thoroughly elucidated yet [8,17]. Studies on the correlation of proteinuria and ocular changes in patients with pre-eclampsia are insufficient. In this study, the authors evaluated the correlation between proteinuria and ocular images using OCT and OCT-A in patients with pre-eclampsia.

## Materials and methods

### Study population

In this retrospective study, 61 patients who were diagnosed with pre-eclampsia and referred to the ophthalmology department during the hospitalisation period from July 2017 to May 2020 were enrolled. Patients who were unable to undergo ophthalmologic and obstetrical evaluation and who had any ocular surgery were excluded. This study followed the tenets of the Declaration of Helsinki and was approved by the Institutional Review Board of Keimyung University Dongsan Hospital, Daegu, Korea (approval number: 2018-06-002). All data were fully anonymised before we accessed them and the Institutional Review Board waived the requirement for an informed consent.

Systolic and diastolic blood pressures (BPs) were measured on admission and ophthalmologic examination. Weight and height of the patient on admission were also measured and body mass index (kg/m^2^) was calculated. Multifetal gestation and obstetrical history and previous illness history was investigated. Urine protein, creatinine and albumin concentrations and serum creatinine, albumin, lactate dehydrogenase, aspirate aminotransferase and alanine aminotransferase concentrations were measured. The injection of intravenous magnesium (Magunesin®, Daewon, Seoul, Korea) and use of blood pressure-lowering agents, such as oral nifedipine (Adalat®, Bayer AG, Leverkusen, Germany) and intravenous hydralazine (Hydralazine HCl®, Samjin, Seoul, Korea), were investigated. All patients were referred to the ophthalmology department 2 days after admission.

Pre-eclampsia was diagnosed according to the criteria agreed by the National High Blood Pressure Education Programme Working Group of National Institutes of Health. Pre-eclampsia was defined as blood pressure of at least 140/90 mmHg after 20 weeks of gestation in a woman with previous normal blood pressure and presence of proteinuria (≥300 mg/24 h).

### Image acquisition and analysis

Ophthalmologic examination includes best-corrected visual acuity, intraocular pressure using Goldmann applanation tonometry (AT 900®, Haag-Streit, Koniz, Germany), refractive error and slit-lamp examination of the anterior and posterior segments. OCT and OCT-A images were obtained using SS-OCT (DRI OCT Triton®, Topcon, Tokyo, Japan) by one skilled examiner. All OCT scans were performed in the afternoon (12:00 pm to 5:00 pm) to avoid diurnal variations of choroidal status [18,19]. Using the thickness map of the macula from raster scan, the average thicknesses of the ganglion cell layer+ (GCL+), GCL++ and choroid in the Early Treatment Diabetic Retinopathy Study (ETDRS) subfield area were automatically calculated. GCL+ is the same concept to ganglion cell-inner plexiform layer; GCL++ consists of three innermost retinal layers (nerve fibre layer, GCL and inner plexiform layer), known as ganglion cell complex [20].

Choroidal vascularity index (CVI) was calculated to explore vascular regions in the choroid from transfoveal horizontal OCT scans according to the method suggested by Agrawal et al. [21].

In 3.0 × 3.0-mm macular scanning OCT-A, the ‘en face’ images were automatically segmented to the superficial capillary plexus (SCP) and deep capillary plexus (DCP). The area measurement tool equipped in IMAGEnet 6 (version 1.22, Topcon, Tokyo, Japan) was used to delineate foveal avascular zone (FAZ); one retinal specialist (JKL) drew a borderline of avascular zone in the superficial and deep retinal vascular images; the area was automatically calculated. The VD (ratio of the area of vessel and microvasculature to the total area) in ETDRS subfields was generated from SCP and DCP images of IMAGEnet 6 using an automated software algorithm. In ETDRS subfields, a 1.0-mm-diameter circle was defined as the central area; the annular area that remained after subtraction of the central area from the 3.0-mm-diameter circle was defined as the paracentral area; paracentral areas were divided into four areas: temporal, nasal, superior and inferior.

### Statistical analysis

To evaluate the relationship between ocular measurement and PCR, according to the median value of PCR (1.35 mg/mg), patients were divided into two groups: group 1 (≥1.35 mg/mg) and group 2 (<1.35 mg/mg). The linear relationship with ocular measurement value was explored after converting the PCR, applying logarithm transformation because the PCR values were skewed.

SPSS version 20.0 for Windows (IBM Co., Armonk, NY, USA) was used for performing statistical analysis including independent Student’s t-test and Pearson tests. Measurements from OCT and OCT-A images of the two groups were compared using independent Student’s t-test. The influence of variable factors on choroidal thickness (CT) was examined using Pearson tests. Path analysis was performed using ‘lavaan’ and ‘semPlot’ packages in R3.6.0 (Copyright (C) 2019 The R Foundation for Statistical Computing Platform). A *p*-value < 0.05 was considered statistically significant.

## Results

The average age of the 61 enrolled patients was 34.3 years. Intravenous magnesium was injected to 20 patients to prevent epilepsy events. Oral or intravenous blood pressure-lowering agents were administered to 46 patients to control increased blood pressure. Moreover, 31 patients belonged to group 1 and 30 to group 2. Systolic BP and use of intravenous magnesium were significantly high in the group with high PCR (Table 1).

**Table 1:** Demographical and clinical features of pregnant women with pre-eclampsia included in the study.

	Group 1 (n = 31)	Group 2 (n = 30)	*p*-value*
Age (years)	35.3 ± 4.4	33.2 ± 4.1	0.062
Right eye BCVA (LogMAR)	0.08 ± 0.15	0.08 ± 0.09	0.936
Left eye BCVA (LogMAR)	0.09 ± 0.16	0.13 ± 0.17	0.363
Right eye IOP (mmHg)	14.3 ± 2.9	14.9 ± 3.8	0.506
Left eye IOP (mmHg)	14.4 ± 2.3	15.4 ± 3.6	0.230
Right eye SE (D)	−2.1 ± 3.0	−2.2 ± 2.3	0.936
Left eye SE (D)	−2.1 ± 2.7	−2.1 ± 2.5	0.936
Body mass index, (kg/m^2^)	29.9 ± 6.2	28.0 ± 6.6	0.263
Gestational age at delivery (weeks)	33.2 ± 4.0	33.0 ± 3.1	0.821
PMA (weeks)	30.0 ± 5.7	31.3 ± 4.4	0.313
Initial SBP (mmHg)	148.1 ± 21.5	158.3 ± 16.6	0.042
Initial DBP (mmHg)	91.3 ± 14.5	97.3 ± 11.1	0.074
SBP on exam (mmHg)	136.9 ± 15.2	140.2 ± 14.8	0.395
DBP on exam (mmHg)	83.2 ± 10.5	86.5 ± 9.2	0.200
Magnesium use (%)	19.4	46.7	0.046
BP-lowering agent use (%)	64.5	86.7	0.716
Twins (%)	16.1	3.3	0.155

*P-value was calculated using independent t-test or Pearson chi-square test.

BCVA, best-corrected visual acuity; IOP, intraocular pressure; SBP, systolic blood pressure; DBP, diastolic blood pressure; SE, spherical equivalent; PMA, postmenstrual age; OD, oculus dexter; OS, oculus sinister; D, diopter.

CT in group 1 was statistically greater than that in group 2, except the inferior and central areas in the left eye. VD and FAZ in the superficial and deep retina, CVI, GCL+ and GCL++ showed no difference between the two groups (Table 2).

**Table 2:** Choroidal and retinal vascularity profile in pregnant women with pre-eclampsia.

		Group 1 (n = 31)	Group 2 (n = 30)	*p*-value*
OD	CVI	0.7 ± 0.0	0.7 ± 0.0	0.876
	CT (C)	232.2 ± 71.7	194.7 ± 60.8	**0.031**
	CT (T)	237.0 ± 63.6	197.1 ± 57.1	**0.012**
	CT (N)	217.1 ± 61.9	181.0 ± 61.9	**0.026**
	CT (S)	237.0 ± 61.0	199.3 ± 59.5	**0.018**
	CT (I)	229.2 ± 54.3	190.7 ± 59.7	**0.011**
	GCL++ (C)	46.4 ± 7.9	49.7 ± 16.9	0.336
	GCL++ (T)	106.8 ± 8.7	106.1 ± 8.2	0.745
	GCL++ (N)	112.5 ± 11.4	112.5 ± 10.7	0.986
	GCL++ (S)	116.2 ± 10.5	117.3 ± 12.4	0.705
	GCL++ (I)	118.3 ± 10.2	117.4 ± 10.3	0.729
	GCL+ (C)	41.2 ± 6.1	43.1 ± 12.7	0.459
	GCL+ (T)	84.9 ± 7.5	84.2 ± 6.9	0.677
	GCL+ (N)	87.7 ± 9.7	85.5 ± 12.6	0.465
	GCL+ (S)	88.3 ± 8.0	88.5 ± 9.5	0.924
	GCL+ (I)	88.9 ± 7.8	87.5 ± 6.8	0.485
	Superficial VD (C)	19.8 ± 4.6	20.8 ± 8.9	0.567
	Superficial VD (T)	48.8 ± 2.7	47.6 ± 3.8	0.163
	Superficial VD (N)	48.9 ± 2.9	48.5 ± 3.5	0.610
	Superficial VD (S)	51.5 ± 5.4	49.5 ± 4.8	0.125
	Superficial VD (I)	51.6 ± 4.5	51.9 ± 4.3	0.797
	Deep VD (C)	17.2 ± 5.8	17.7 ± 1.0	0.807
	Deep VD (T)	50.1 ± 3.5	50.0 ± 4.6	0.922
	Deep VD (N)	51.8 ± 4.3	51.6 ± 4.6	0.859
	Deep VD (S)	52.3 ± 5.8	52.7 ± 4.1	0.753
	Deep VD (I)	56.4 ± 3.7	56.4 ± 5.6	0.993
	Superficial FAZ	304.7 ± 100.2	309.0 ± 125.8	0.882
	Deep FAZ	387.2 ± 134.8	455.3 ± 174.3	0.094
OS	CVI	0.7 ± 0.0	0.7 ± 0.1	0.702
	CT (C)	230.6 ± 48.4	200.4 ± 68.3	0.051
	CT (T)	233.8 ± 45.6	205.6 ± 58.1	**0.040**
	CT (N)	215.7 ± 52.0	182.5 ± 66.9	**0.035**
	CT (S)	228.0 ± 49.6	187.2 ± 64.2	**0.008**
	CT (I)	229.8 ± 55.6	204.4 ± 64.6	0.106
	GCL++ (C)	44.0 ± 8.1	50.8 ± 23.2	0.131
	GCL++ (T)	106.6 ± 8.3	106.1 ± 7.9	0.810
	GCL++ (N)	113.2 ± 10.4	116.2 ± 14.3	0.349
	GCL++ (S)	116.3 ± 9.4	116.3 ± 10.2	0.997
	GCL++ (I)	118.8 ± 9.3	116.8 ± 10.6	0.423
	GCL+ (C)	39.2 ± 6.6	41.5 ± 9.6	0.263
	GCL+ (T)	85.0 ± 7.3	83.4 ± 8.9	0.461
	GCL+ (N)	88.5 ± 8.7	88.0 ± 12.1	0.844
	GCL+ (S)	88.9 ± 7.2	87.2 ± 8.7	0.408
	GCL+ (I)	89.1 ± 7.3	86.6 ± 11.6	0.312
	Superficial VD (C)	18.0 ± 3.0	19.9 ± 7.2	0.175
	Superficial VD (T)	50.6 ± 3.9	50.3 ± 3.3	0.707
	Superficial VD (N)	47.7 ± 3.4	47.0 ± 3.2	0.405
	Superficial VD (S)	51.4 ± 4.1	50.6 ± 3.1	0.412
	Superficial VD (I)	52.9 ± 3.1	52.4 ± 5.7	0.719
	Deep VD (C)	15.1 ± 4.0	18.1 ± 9.5	0.112
	Deep VD (T)	52.1 ± 4.0	50.8 ± 4.7	0.254
	Deep VD (N)	49.2 ± 3.7	49.5 ± 4.2	0.742
	Deep VD (S)	54.0 ± 4.0	54.0 ± 4.2	0.946
	Deep VD (I)	58.5 ± 3.2	54.7 ± 5.7	**0.003**
	Superficial FAZ	313.6 ± 102.8	295.9 ± 124.3	0.548
	Deep FAZ	429.7 ± 138.8	402.3 ± 133.4	0.440

*P-value was calculated using independent t-test.

CVI, choroidal vascularity index; CT, choroidal thickness; C, central; T, temporal; N, nasal; S, superior; I, inferior; GCL, ganglion cell layer; VD, vascular density; FAZ, foveal avascular zone; OD, oculus dexter; OS, oculus sinister.

Central CT (*r* = 0.284, *p* = 0.026) showed significant linear relationship with PCR after logarithm transformation. Other ocular factors failed in demonstrating significant relationship with PCR. The association between CT and CVI was not observed. The mean arterial pressure (MAP) showed significant linear relationship with PCR after logarithm transformation (*r* = 0.296, *p* = 0.021), but there was no significant relationship with other ocular factors (Table 3) (Fig 1)

**Fig 1:** Correlations among logPCR, CT, MAP and CVI. (A–C) logPCR correlations with CT, MAP and CVI with a linear fit line. (D) CVI correlation with CT with a linear fit line. Correlation values are (A) *r* = 0.284, *p* = 0.026, (B) *r* = 0.296, *p* = 0.021, (C) *r* = −0.083, *p* = 0.527 and (D) *r* = 0.023, *p* = 0.858. CT, choroidal thickness; logPCR, protein–creatinine ratio in urine after logarithm transformation; CVI, choroidal vascularity index; MAP, mean arterial pressure.

**Table 3:** Ocular factors associated with logPCR, CT and MAP.

	**logPCR**		**CT**		**MAP**	
	Coefficient (*r*)	*p*-value*	Coefficient (*r*)	*p*-value*	Coefficient (*r*)	*p*-value*
**logPCR**	-	-	0.284	0.026	0.296	0.021
**CVI**	−0.083	0.527	0.023	0.858	-.0.026	0.844
**CT (C)**	0.284	0.026	-	-	0.050	0.704
**GCL++ (C)**	−0.181	0.162	0.210	0.105	−0.052	0.957
**GCL+ (C)**	−0.149	0.252	0.156	0.233	−0.058	0.986
**Superficial VD (C)**	−0.077	0.554	−0.157	0.228	0.080	0.542
**Deep VD (C)**	−0.082	0.532	−0.166	0.201	0.048	0.715
**Superficial FAZ**	0.097	0.457	−0.247	0.055	0.115	0.378
**Deep FAZ**	−0.021	0.872	−0.249	0.053	0.052	0.691

*P-values and correlation coefficients (*r*) were calculated using parametric correlation analysis.

MAP, mean arterial pressure; logPCR, protein–creatinine ratio in urine after logarithm transformation; CVI, choroidal vascularity index; CT, choroidal thickness; C, central; GCL, ganglion cell layer; VD, vascular density; FAZ, foveal avascular zone.

The path analysis disproved the model in which MAP acts as an intermediary variable between PCR and CT (χ^2^ = 5.193, *p* = 0.023) and revealed that the model that postulates a direct causal relationship between PCR and CT was valid (χ^2^ = 0.704, *p* = 0.144) (Fig 2).

**Fig 2:** Path analysis of logPCR, MAP and CT. Path coefficients (values adjacent to the arrow) correspond to the standardised coefficients calculated via the analysis of correlation matrices. (A) Structured model. Significant relations were observed between PCR and CT and PCR and MAP but not MAP and CT. (B) Model in which MAP act as an intermediary variable was invalid (χ^2^ = 5.193, df = 1, *p* = 0.023), (C) Model that postulates a direct causal relationship between PCR and CT was valid (χ^2^ = 0.704, *p* = 0.144). CT, choroidal thickness; logPCR, protein–creatinine ratio in urine after logarithm transformation; MAP, mean arterial pressure.

## Discussion

Vascular changes in patients with pre-eclampsia occur systematically. Systemic vasoconstriction is caused by various factors, including the upregulated formation of endothelium and superoxide; decreased formation of vasodilators (such as nitric oxide) and increased vascular sensitivity to angiotensin II. Multiorgan failure follows endothelial dysfunction and hyperpermeability, causing cytotoxic and vasogenic oedema [22]. The choroid is more sensitive to changes of pre-eclampsia than other organs due to its high VD, fenestrated capillaries and autonomic nerve controls. It was demonstrated that the choroid was responsive to circulating angiogenic factors, such as soluble endoglin (sEng), placental growth factor (PlGF) and VEGF [23,24]. Stern-Ascher et al. [8] found a positive association of PlGF with central CT in severe pre-eclampsia, suggesting that intravascular inflammation and vasoconstriction caused by pre-eclampsia does affect CT. In the study comparing CT among three groups of normotensive non-gravid, normotensive postpartum and pre-eclampsia postpartum women using EDI OCT, Garg et al. [9] reported that pre-eclampsia postpartum cases had greater CT and retinal macular volume than normotensive postpartum without difference of these values between normotensive postpartum and normotensive non-gravid women and suggested that it was due to higher serum-VEGF concentration in pre-eclampsia patients than normotensive pregnant women, which was reported by Celik at al. [10]. Similarly, Kim et al. [25] also reported increased CT in patients with pre-eclampsia, but normal CT in healthy pregnant patients.

In patients with pre-eclampsia, vascular endothelial function is damaged, which increases permeability of the glomerular basement membrane against serum proteins and albumins [26]. Proteinuria caused due to increased permeability of the glomerulus is an important diagnostic criteria of pre-eclampsia. Dong et al. revealed that proteinuria in patients with pre-eclampsia is closely related to disease severity [27]. PCR is a simple, inexpensive and easily accessible method to assess the magnitude of proteinuria and the function of glomerular cell [16,28,29]. In this study, CT was significantly increased with elevated PCR. These results imply that choroidal changes in patients with pre-eclampsia possibly represent not only ocular condition but also systemic vascular state. Garg et al. [9] suggested that, considering the fact that circulating angiogenic factor level closely related to CT increases 5 weeks before the onset of clinical symptoms of pre-eclampsia, it is plausible to use CT as a predictive marker for pre-eclampsia. Considering our study implied the close relationship between CT and PCR, CT may play a role as a predictive and quantitative marker of pre-eclampsia.

CVI is an emerging quantitative biomarker of CT [21,30–32]. Reportedly, CVI was higher in patients with acute central serous chorioretinopathy (CSCR) than in control groups and decreased as CSCR resolved [31]. Tan et al. [30] mentioned that a decrease in CVI was observed in patients with diabetes mellitus than in age-matched control groups. The use of CVI as a marker of disease activity in patients with inflammatory chorioretinal pathology was raised by researchers [33,34]. In our study, CVI was not significantly associated with PCR or CT. This suggests that dilatation and increased permeability of choroidal vasculature in pre-eclampsia lead to an increase in both luminal and stromal spaces with similar rate.

There are still some controversies on whether pre-eclampsia affects the retina. In the literature, Kim et al. [25] and Ciloglu et al. [35] reported no significant increase in central subfield retinal thickness among groups of healthy pregnancy, pregnancy with pre-eclampsia and non-pregnancy. Demir et al. [36] found that parafoveal retinal thickness was greater in healthy pregnant women than that in control groups and reported that fluid retention caused by hyperpermeability of vessels increases thickness of the retina. Demir et al. also found that there was no significant difference in terms of foveal retinal thickness among the above-mentioned groups. In contrast, Atas et al. [37] showed that the foveal retinal thickness was less in women with pre-eclampsia and healthy pregnant women than that in healthy non-pregnant women. Neudorfer et al. [14] and Ciloglu et al. [35] reported increased peripapillary retinal nerve fibre layer thickness in pregnancy with pre-eclampsia. This study did not show any association of PCR and the thickness of GCL++ and GCL+ in the macular region. We speculate two reasons. First, that systemic hyperpermeability and endothelial dysfunction had less effect on the retinal tissue than on the choroidal tissue because the retinal vasculature has autoregulation and lower density than that of the choroid. Second, blood pressure in this study was not high enough to induce hypertensive retinopathy from blood pressure-lowering agents.

FAZ is an area devoid of retinal capillaries. Recently, the evaluation of clinical correlation and response to treatment via FAZ using OCT-A in diabetic macular oedema and branched retinal vein occlusion has been attempted [38–40]. Ciloglu et al. [35] investigated FAZ and VD of SCP and DCP using OCT-A in groups of pregnancy with pre-eclampsia, healthy pregnancy and non-pregnancy. There was no significant difference in FAZ among the groups; however, VD of DCP was more susceptible in groups of pregnancy with pre-eclampsia. They revealed that DCP was more influenced by generalised vasospasm due to its high metabolic activity and complex structure. The present study showed no association of PCR with FAZ and VD of the SCP or DCP. In patients with pre-eclampsia, two cardiovascular changes happen simultaneously. One is systemic vascular constriction. In normal pregnancy, systemic vasodilatation accompanies decrease in blood pressure. However, pregnant women with pre-eclampsia have impaired endothelial function, which triggers systemic vasoconstriction and increases peripheral vascular resistance [41,42]. Lupus et al. [43] reported that systemic vasoconstriction of pregnant women with pre-eclampsia leads to constriction of the retinal microvasculature. The other is systemic hypertension, which is caused by enhanced angiotensin II sensitivity accompanied by vasoconstriction through activation of endothelin-1 [26,44]. We speculate that, although vasospasm interrupts blood flow in the retina, hydrostatic pressure of blood compensates this obstacle, whereas endothelial dysfunction has little influence on blood flow in the retina. We also suggest that long-term severe pre-eclampsia may induce changes in retinal thickness and vasculature similar to hypertensive retinopathy.

Pathologic fundus findings in patients with pre-eclampsia include optic neuropathy, retinal haemorrhages, Elschnig’s spots, cotton wool spots, segmental or generalised vasoconstriction and serous retinal detachment, which are also commonly found in hypertensive retinopathy [7]. Previously, high blood pressure itself was considered the main cause of chorioretinopathy of patients with pre-eclampsia. However, many studies have expressed doubt on that idea. Gupta et al. [45] and Gooding et al. [17] reported that high blood pressure does not have an impact on retinal thickness. Iwase et al. [46] suggested the positive relationship of CT and blood pressure but also admitted that it was insufficient to support the idea that increase or decrease in blood pressure was the direct cause of changes in CT. In the study of Kim et al. [25], accumulation of sub-retinal fluid was observed in seven patients. The authors suggested that the cause of sub-retinal fluid accumulation was increased hydrostatic pressure due to choroidal thickening, not hypertensive retinopathy. In this study, MAP showed significant association with PCR but no significant association with chorioretinal factors (GCL, FAZ, VD, CT, CVI). The path analysis showed that PCR may directly act on CT, not through an influence on MAP. When the two different models were compared, the model that postulates a direct causal relationship between PCR and CT was found to fit the data, whereas the other model in which PCR acts on CT through an influence on MAP was found to be invalid (Fig 2).

Considering these results, we offer two suggestions. First, that chorioretinal pathology and hypertension are independent results of systemic imbalance. Our results showed that hypertension was not related to ocular changes, which conflicts with the previous idea that pathologic ocular findings in pre-eclampsia are induced by hypertension. We may speculate that although systemic imbalance of vascular factors affects both blood pressure and ocular vascular condition, progression to a pathologic occurs independently. Second, we suggest that the previously established model, in which chorioretinal changes in pre-eclampsia are attributed to hypertensive chorioretinopathy, should be replaced with a model that postulates chorioretinal changes primarily arising from pre-eclampsia vascular pathology. Thus, ‘pre-eclampsia chorioretinopathy’ would be a more appropriate term.

This study has several limitations. The choroid is an organ sensitive to hormonal situations and gestational age (GA) [9,47,48]. Accordingly, the average CT can be different in each stage. The small sample size may have insufficient significance to explain the relationship. Participants of this study underwent ophthalmologic examination as soon as they were referred to the ophthalmology department; however, some patients underwent ocular evaluation after the start of treatment, such as BP control, which impeded the exact evaluation of the relationship between BP and ocular factors. Patients whose condition was too poor to undergo OCT and OCT-A were excluded.

In conclusion, CT in pre-eclampsia is correlated with PCR, implying pre-eclampsia severity. Furthermore, this study makes us reconsider the idea that ocular complications in patients with pre-eclampsia are derived from hypertension but are rather caused by systemic vascular changes in pre-eclampsia.
